This article has been retracted.

# Effects of Dexmedetomidine Combined with Intravenous Anesthesia on Oxidative Stress Index, Postoperative Sleep Quality, and Brain Function in HICH Patients

**DOI:** 10.1155/2022/5463986

**Published:** 2022-03-19

**Authors:** Jiong Shi, Guangping Zhao, Panpan Liu, Yuwei Bai, Yongxue Chen

**Affiliations:** Anesthesiology Department, Handan Central Hospital, Handan 056001, China

## Abstract

To investigate the effects of dexmedetomidine combined with intravenous anesthesia on oxidative emergency indicators, postoperative sleep quality, and brain function in patients with hypertensive cerebral hemorrhage (HICH), a total of 285 HICH patients admitted to our hospital from February 2020 to February 2021 were selected. The combined anesthesia group (*n* = 142) and the control group (*n* = 143) were established by the random number table method. The control group received conventional intravenous anesthesia, and the combined anesthesia group received dexmedetomidine combined intravenous anesthesia. Two groups of patients before and after operation was observed vital signs, oxidative stress index difference, comparing each time, the change of the two groups of brain function index, adverse reactions occurred between observation group, and the postoperative period of Pittsburgh Sleep Quality Index Scale (PSQI) score as a result, the Pearson correlation coefficient analysis of oxidative stress level and the correlation of HICH patients sleep quality. After operation, the mean arterial pressure (MAP) and heart rate (HR) of patients in both groups decreased significantly. The MAP level in the combined anesthesia group significantly increased compared to the control group, and the HR level decreased significantly than the control group (all *P* < 0.05). The levels of TNF-*α*, IL-6 and MDA in both groups increased significantly on day 7 after operation compared with before operation, but the indexes in the combined anesthesia group significantly decreased compared with the control group (*P* < 0.05). The level of superoxide dismutase (SOD) in both groups significantly decreased compared to that before operation, and the index value in combined anesthesia group significantly increased compared to that in the control group (*P* < 0.05). After surgery, the levels of central nerve specific protein (S100-*β*) and neuron specific enolase (NSE) in 2 groups increased with time, and the indexes in the combined anesthesia group significantly decreased compared to the control group (all *P* < 0.05). The incidence of adr in combined anesthesia group decreased significantly than that in control group (*P* < 0.05). After surgery, PSQI scores of the two groups showed a downward trend with time extension, and scores of the combined anesthesia group decreased significantly than those of the control group at 24 h, 48 h and 7 d after surgery (all *P* < 0.05). Pearson's correlation coefficient was used to analyze that TNF-*α*, IL-6, and MDA levels were positively correlated with PSQI score, while SOD level was negatively correlated with PSQI score (all *P* < 0.05). Dexmedetomidine combined with intravenous anesthesia can significantly improve the vital signs and oxidative stress response of HICH patients, effectively reduce the risk of adverse reactions, have little impact on the brain function of patients, and can improve the postoperative sleep quality of patients. This operation is worthy of clinical application. In addition, this study further analyzed the influence mechanism of postoperative sleep quality in patients with HICH and showed that TNF-*α*, IL-6, MDA, and SOD were all correlated with sleep quality in patients with HICH, suggesting that follow-up detection of these indicators has positive significance in improving the prognosis of patients.

## 1. Introduction 

Hypertensive cerebral hemorrhage is a type of severe complication in the disease of heart head blood-vessel. Its onset mechanism for patients with chronic hypertension or blood pressure significantly causes brain artery lesions and causes blood vessel burst bleeds. A large number of intracranial hematomas occur in patients [1]. If the diagnosis and treatment are not made in time, the amount of intracranial hematoma will be further aggravated and the life safety of patients will be seriously affected [2]. At the present stage, surgical treatment is mostly carried out for HICH patients, but the final surgical effect is susceptible to the effects of anesthesia and anesthesia effects, and considering the characteristics of patients' clinical conditions and the particularity of the surgical site, intraoperative anesthesia control and management are more difficult [3]. Scientific anesthesia management is an important guarantee to improve the surgical effect and prognosis of patients in clinical practice. At present, there are a lot of clinical applications of general anesthetic propofol with anesthesia and visible effects quickly. The advantages of the analgesic effect are good, but the drug propofol has an inhibitory effect on the cardiovascular system, and continuous or static notes easily cause hemodynamics in patients with excessive imbalances, increased stress damage, brain surgery, and postoperative may affect patients' sleep quality, and it is not conducive to the rapid recovery of brain function [4]. Dexmedetomidine is a new class of *α* 2-adrenergic receptor agonists with significant efficacy, which has a positive effect on reducing sympathetic nerve activity and plasma cortisol concentration, suggesting that it can relieve central nerve injury symptoms and protect brain function in patients to a certain extent [5]. At present, there are few reports about the application of dexmedetomidine combined with intravenous anesthesia in emergency HICH patients, and its clinical advantages are still unclear. Based on this, this study explored the effects of dexmedetomidine combined with intravenous anesthesia on oxidative stress indicators, postoperative sleep quality, and brain function of HICH patients and analyzed the relevant mechanisms in depth in order to provide clinical reference.

The rest of this paper is organized as follows.  Section 2 summarizes data and methods and related studies. In Section 3, the experimental results are given in detail. The discussion is presented in Section 4. Conclusion and future work are summarized in Section 5.

## 2. Data and Methods

### 2.1. General Data

A total of 285 HICH patients admitted to our hospital for treatment from February 2020 to February 2021 were selected, and a combined anesthesia group (*n* = 142) and control group (*n* = 143) were established according to the random number table method. In the combined anesthesia group, there were 79 males and 63 females, aged from 34 to 70 years old, with an average of 58.17 ± 6.43 years old. The body mass index (BMI) was 18.62–26.08 kg/m^2^, with an average of 23.64 ± 1.52 kg/m^2^. The Glasgow Coma Scale (GCS) at admission ranged from 6 to 12 points, with an average of 9.84 ± 2.03. In the control group, there were 75 patients, including 68 females, aged from 37 to 72 years old, with an average of 56.91 ± 5.72 years old. The BMI ranged from 18.53 to 25.97 kg/m^2^, with an average of 23.39 ± 1.47 kg/m^2^. The GCS score was 7–13 points, with an average of 10.02 ± 2.11 points. There were no significant differences in gender, age, BMI, GCS score, and other general data between the two groups (*P* > 0.05). It was confirmed that the comparison between groups was scientifically reasonable. The inclusion criteria were as follows: (1) all patients with a history of hypertension who had their first attack of HICH; (2) the interval from onset to hospitalization was less than 12 h; (3) no other relevant treatment plan was received before admission to our hospital; (4) rated as II–III by the American Society of Anesthesiologists, ASK [6]; (5) the Athens Insomnia Scale (AIS) ≤6 points [7]; and (6) the clinicopathological data were complete, and the patients and their families understood the study and gave informed consent. The exclusion criteria were as follows: (1) patients with severe infection, severe blood disease, malignant tumor disease, or immune system disease at admission; (2) complicated with serious organic diseases such as liver and kidney; (3) contraindications or allergies of the drugs used in this study; and (4) patients with a history of chronic sedative and analgesic drugs.

### 2.2. Methods

#### 2.2.1. Operation and Anesthesia Methods

Craniotomy was performed for patients in both groups. Before surgery, patients were given 0.5 mg of atropine and 100 mg of phenobarbital sodium 30 min before surgery. Intramuscular injection was adopted. After entering the operating room, intravenous access was established and oxygen inhalation was given by masks. The control group was injected with 0.9% sodium chloride solution, and the combined anesthesia group was pumped with dexmedetomidine 0.5 *μ*g/kg (Jiangsu Nhwa Pharmaceutical Co., Ltd.; national drug approval number H20110085; specification: 2 mL: 0.2 mg). The pumping time was controlled within 10 min, and then maintained at 0.5 *μ*g/kg·H-1. Anesthesia induction drugs for all patients were atracurium 0.2 *μ*g/kg, sufentanil 0.3 *μ*g/kg, and propofol 2 mg/kg. After tracheal intubation, the patients were connected to a ventilator, CO2 partial pressure at the end of expiratory was set to 30–35 mmHg (1 mmHg = 0.133 kpa), respiration rate was 12 times/min, and propofol pump was maintained. The velocity was adjusted appropriately according to the patient's hemodynamic changes and intraoperative conditions. Atracurium 0.03 mg/kg was added at 30 min intervals, and the patient's heart rate and blood pressure were treated appropriately. Sufentanil infusion was stopped 30 min before the end of surgery, dexmedetomidine infusion was stopped 15 min before the end of surgery, and propofol pump infusion was stopped when the skin suture was about to be completed.

### 2.3. Index Detection Methods

5 mL of fasting venous blood was taken from patients before and after surgery, centrifuge parameters were set to 3500 r/min, centrifuge radius was 10 cm, centrifuge time was 10 min, and supernatant was taken. Brain function indexes including S100-*β* and NSE were determined by enzyme-linked immunosorbent assay (ELISA). The oxidative stress indexes including tumor necrosis factor *α* (TNF-*α*), interleukin-6 (IL-6), and malondialdehyde (malondialdehyde) were also measured by the abovementioned serum samples, and the specific indexes included tumor necrosis factor *α* (TNF-*α*), interleukin-6 (IL-6), malondialdehyde (MDA), and superoxide dismutase (SOD).

### 2.4. Indicators

1. The difference in vital signs between the two groups before and after surgery was compared, including oxygen saturation (SpO2), mean arterial pressure (MAP), and heart rate (HR); (2) comparison of oxidative stress indexes between the two groups before and after surgery; (3) the differences in brain function indexes at different time periods between the two groups were compared, including S100-*β* protein and NSE indexes before surgery, immediately after surgery, 6 h, 12 h, and 24 h after surgery; (4) adverse reactions were compared between the two groups, including agitation, hypotension, tachycardia, bradycardia, nausea, and vomiting; (5) the PSQI scores of the two groups at each time point after surgery were compared, including the scores at 24 h, 48 h, and 7 d after surgery; (6) Pearson's correlation coefficient was used to analyze the correlation between the oxidative stress index level and sleep quality of HICH patients.

### 2.5. Evaluation Criteria of Sleep Quality

The Pittsburgh Sleep Quality Index (PSQI) was used to evaluate the sleep quality of patients at 24 h, 48 h, and 7 d after surgery [8]. The total score of the PSQI was 21 points, and the sleep quality of patients decreased with the increase of the score. A score of less than or equal to 5 indicates very good sleep quality, 6 to 10 indicates good sleep quality, 11 to 15 indicates fair sleep quality, and 16 to 21 indicates poor sleep quality.

### 2.6. Statistical Methods

The data was sorted, and the database was established. The SPSS 26.0 software was used for statistical analysis of all the data. The measurement data to normality and the f test met the normal distribution; the mean ± standard deviation ($\bar{x}$ ± *s*) determined the group row data differences between two independent sample *t*-tests and paired *t*-tests; counting data use (%) determined the *x*^2^ square test. Repeated measures OVA were used for data at different time points in the group, and the Mauchly test was used for data comparison. *P* > 0.05 indicated full football symmetry of covariance. Pearson's correlation coefficient was used to analyze the correlation between the oxidative stress index level and sleep quality of HICH patients, and *P* < 0.05 proved to be statistically significant.

## 3. Results

### 3.1. Comparison of Vital Signs Differences

There was no significant difference in the level of SpO2 between groups (all *P* < 0.05); there were no statistically significant differences in MAP and HR indexes before surgery (*P* > 0.05), and the levels of both indexes decreased significantly after surgery. The MAP level in the combined anesthesia group significantly increased compared to the control group, while the HR level significantly decreased compared to the control group (all *P* < 0.05).  Table 1 shows the comparison of vital signs.

### 3.2. Comparison of Oxidative Stress Indexes

Before surgery, there were no significant differences in the levels of indexes between 2 groups (all *P* > 0.05). The levels of TNF-*α*, IL-6, and MDA in both groups increased significantly than those before the operation on 7 days after the operation, and the comparison between groups showed that the levels of TNF-*α*, IL-6, and MDA in the combined anesthesia group decreased significantly than those in the control group (*P* < 0.05). The SOD level in both groups decreased significantly than before 7 days after surgery, and the comparison between groups showed that the SOD level in the combined anesthesia group increased significantly than the control group 7 days after surgery (*P* < 0.05), as shown in Table 2.

### 3.3. Comparison of Brain Function Index Levels

Before surgery, there were no significant differences in S100-*β* protein and NSE index (all *P* > 0.05). After surgery with the extension of time, the levels of all indexes in the two groups were increased, and the levels of S100-*β* protein and NSE indexes in the combined anesthesia group significantly decreased compared to the control group (all *P* < 0.05).  Table 3 shows the comparison of S100-*β* protein levels.  Table 4 presents a comparison of NSE index levels.

### 3.4. The Incidence of Adverse Reactions Was Compared

The incidence of agitation, hypotension, tachycardia, bradycardia, nausea, and vomiting in the combined anesthesia group decreased compared to those in the control group, and the incidence of adverse reactions decreased significantly compared to those in the control group (*P* < 0.05).  Table 5 shows the comparison of adverse reactions.

### 3.5. Comparison of PSQI Scores at Each Time Point

After surgery, the PSQI scores showed a downward trend with the extension of time, and the scores of the combined anesthesia group significantly decreased compared to the control group at 24 h, 48 h, and 7 d after surgery (all *P* < 0.05).  Table 6 shows the differences in PSQI scores at different time points.

### 3.6. Analysis of the Correlation between Oxidative Stress Index Level and Sleep Quality of HICH Patients

Pearson's correlation coefficient was used to analyze that TNF-*α*, IL-6, and MDA levels were positively correlated with PSQI score, while SOD level was negatively correlated with PSQI score (all *P* < 0.05).  Figure 1 shows the correlation between the oxidative stress index level and sleep quality of HICH patients.

Clinical studies have shown that the incidence of HICH has increased significantly in recent years, and adverse symptoms such as secondary cerebral ischemia and hypoxia are common in patients after the onset of HICH, and brain damage will be further caused if the diagnosis and treatment are not enough, which is also an important reason for the poor prognosis of patients [9]. Other literature shows that surgical trauma can affect the inflammatory factors of HICH patients, trigger the occurrence of inflammatory responses in patients, and then activate the release of immune mediators in large quantities, and the serum TNF-*α*, IL-6, and other proinflammatory factors increase significantly, aggravating traumatic brain parenchymal damage and inducing an oxidative stress response in patients [10, 11]. Dexmedetomidine, as a kind of new sedative drug, has been applied in some surgical operations with significant effect, suggesting the feasibility of the application of dexmedetomidine in anesthesia of HICH pa tients.

## 4. The Experimental Analysis

The analysis confirmed that combined anesthesia could help HICH patients maintain a continuous and stable state of hemodynamics and improve cerebral tissue perfusion in HICH patients, similar to the results of [12]. In order to explore the anesthesia surgery in patients with HICH the reaction of oxidative stress, this study aimed at comparing two groups of patients with inflammatory factor index level, TNF alpha showed postoperative combined anesthesia group, IL - 6, index level significantly decreased, confirming that the right supporting microphone set combined intravenous anesthesia operation for HICH patients body inflammatory reaction, has obvious effect. HICH patients are oppressed by intracranial hematoma after onset, resulting in continuous ischemia of normal intracranial tissues, which destroys the balance between oxidative defense and oxygen free radicals and then causes oxidative stress injury [13]. SOD is the main antioxidant substance of the body, which can remove oxygen-free radicals and reduce oxidative stress damage of the body. MDA is a lipid peroxidation product, and its content represents the severity of cell membrane damage by oxygen-free radicals [14, 15]. This contrast between the study groups shows that in the combined anesthesia group the index of MDA level is significantly lower than that of the control group, the SOD level is obviously higher than that of the control group (*P* < 0.05), and analyzing its mechanism may be related to drug ingredients. The beautiful mi set contains ingredients that stimulate patients' locus coeruleus receptors in the brain, further giving play to the role of antianxiety and alleviating patients' stress reactions in the process of operation. In addition, no respiratory or respiratory inhibition effect was found in clinical application of this drug, which has a unique awake sedation effect and reduces the risk of postoperative adverse reactions [16]. S-100*β* protein and NSE indicators are important markers for the evaluation of central nervous system injury and have been widely used in clinical evaluation of brain function [17]. In this study, it was found that with the extension of time, the levels of all indexes in the two groups increased, and the S100-*β* protein and NSE indexes in the combined anesthesia group were significantly lower than those in the control group at each time, indicating that continuous postoperative infusion of dexmedetomidine is beneficial to the recovery of postoperative brain injury, and its clinical application has high safety and effectiveness.

Postoperative sleep disorder is one of the common adverse symptoms of clinical surgical patients, which is manifested by low sleep efficiency, short sleep duration, and other characteristics, which affect the recovery of patients physically and psychologically [18]. In a study of an analgesic drug regimen after hysteromyomectomy, dexmedetomidine was found to have a positive effect on the improvement of sleep efficiency and reduction of the awakening index of such patients [19]. This research adopted the PSQI score of two groups of patients to evaluate the sleep quality. The analysis found the right beauty holds the mi mechanism in the locus coeruleus nuclear receptor alpha 2, can regulate the activity of the locus coeruleus norepinephrine system, the blood flow to the brain caused by the signal blood flow signal is similar to that of a natural, can reduce the patients with cerebral cortical arousal levels, and improve the patients' sleep disorder state of awakening pathways. Thus, sleep quality of patients can be improved [20]. In order to further explore the influencing mechanism of postoperative sleep quality of HICH patients, the Pearson correlation coefficient was analyzed in this study, and the levels of TNF-*α*, IL-6, and MDA were positively correlated with PSQI score, while SOD level was negatively correlated with PSQI score (all *P* < 0.05) [21–23]. It provides monitoring indicators for the rapid postoperative recovery and sleep quality evaluation of follow-up clinical HICH patients and has a high reference value for the follow-up improvement of patient diagnosis and treatment mechanism. But the conclusion remains to be demonstrated for HICH patients' sleep quality and oxidative stress index correlation analysis, yet other scholars have the same idea, so this research result is difficult to have good persuasive, and this study also has certain deficiencies, such as the study sample size being small, the results may appear biased [24, 25]. Therefore, a larger sample size is needed for further research.

## 5. Conclusion

In conclusion, dexmedetomidine combined with intravenous anesthesia has obvious anesthesia efficacy for HICH patients and has positive effects on reducing patients' oxidative stress responses, improving postoperative sleep quality, and improving brain function, which is worthy of clinical application. In addition, this study further analyzed the influence mechanism of postoperative sleep quality in HICH patients, providing reference data for clinical improvement of patient prognosis and improvement of diagnosis and treatment plan.

## Figures and Tables

**Figure 1:** Correlation between the oxidative stress index level and sleep quality of HICH patients.

**Table 1:** Comparison of vital signs ($\bar{x}$ ± *s*).

Group	SpO2 (%)		MAP (mmHg)		HR (times/min)	
	Before the operation	After the operation	Before the operation	After the operation	Before the operation	After the operation
Combined anesthesia group (*n* = 142)	94.68 ± 3.42	95.34 ± 3.49	121.76 ± 8.32	96.74 ± 5.62^*∗*^	85.03 ± 6.26	71.07 ± 5.22^*∗*^
The control group (*n* = 143)	95.07 ± 3.51	96.41 ± 3.60	122.03 ± 8.47	88.69 ± 5.48^*∗*^	84.69 ± 6.14	77.82 ± 5.41^*∗*^
*T*	−0.950	−1.119	−0.271	12.242	0.463	-10.717
*P*	0.343	0.264	0.786	＜0.001	0.644	＜0.001

*Note.* ^*∗*^Comparison with preoperative, *P* < 0.05.

**Table 2:** Comparison of oxidative stress indexes ($\bar{x}$ ± *s*).

Group	TNF-*α* (mg/L)		IL-6 (mg/L)		MDA (mmol/L)		SOD (U/L)	
	Before the operation	7 days after surgery	Before the operation	7 days after surgery	Before the operation	7 days after surgery	Before the operation	7 days after surgery
Combined anesthesia group (*n* = 142)	1.87 ± 0.22	2.75 ± 0.27^*∗*^	2.28 ± 0.19	4.67 ± 0.42^*∗*^	3.75 ± 0.36	6.07 ± 0.44^*∗*^	100.93 ± 10.74	81.43 ± 8.65^*∗*^
The control group (*n* = 143)	1.84 ± 0.19	3.64 ± 0.33^*∗*^	2.31 ± 0.20	6.02 ± 0.53^*∗*^	3.71 ± 0.32	7.83 ± 0.58^*∗*^	102.12 ± 11.18	66.17 ± 7.52^*∗*^
*T*	1.232	−24.908	−1.298	−23.831	0.992	−28.845	−0.916	15.897
*P*	0.219	<0.001	0.195	<0.001	0.322	<0.001	0.360	<0.001

*Note.* ^*∗*^Comparison with preoperative, *P* < 0.05.

**Table 3:** Comparison of S100-*β* protein levels (*μ*g/L, $\bar{x}$ ± *s*).

Group	Before the operation	Immediately after surgery	6 h after surgery	12 h after surgery	24 h after surgery
Combined anesthesia group (*n* = 142)	0.21 ± 0.06	1.54 ± 0.47^*∗*^	1.71 ± 0.62^∗#^	1.92 ± 0.69^∗#&^	2.01 ± 0.32^∗#&^
The control group (*n* = 143)	0.22 ± 0.05	2.23 ± 0.54^*∗*^	2.59 ± 0.71^∗#^	2.77 ± 0.74^∗#&^	2.96 ± 0.34^∗#&Δ^
*t*	−1.529	−11.503	−11.142	−10.027	−24.286
*P*	0.127	<0.001	<0.001	<0.001	<0.001
Between groups	*F* = 5.672, *P*=0.000				
Different points in time	*F* = 5.154, *P*=0.000				
Between groups *·* different time points	*F* = 4.741, *P*=0.000				

*Note.* ^*∗*^Comparison with preoperative, *P* < 0.05; ^#^Comparison with immediately after surgery, *P* < 0.05; ^&^Comparison with 6 h after surgery, *P* < 0.05; ^△^Comparison with 12 h after surgery, *P* < 0.05.

**Table 4:** Comparison of NSE index levels (ng/mL, $\bar{x}$ ± *s*).

Group	Before the operation	Immediately after surgery	6 h after surgery	12 h after surgery	24 h after surgery
Combined anesthesia group (*n* = 142)	9.12 ± 1.24	9.84 ± 1.31^*∗*^	10.29 ± 1.56^∗#^	10.52 ± 1.61^∗#^	10.67 ± 1.72^∗#^
The control group (*n* = 143)	9.06 ± 1.08	10.52 ± 1.36^*∗*^	11.05 ± 1.73^∗#^	11.87 ± 1.84^∗#&^	14.26 ± 2.11^∗#&Δ^
*T*	0.436	−4.298	−3.894	−6.590	−15.737
*P*	0.663	<0.001	<0.001	<0.001	<0.001
Between groups	*F* = 5.351, *P*=0.000				
Different points in time	*F* = 5.134, *P*=0.000				
Between groups *·* different time points	*F* = 5.012, *P*=0.000				

*Note.* ^*∗*^Comparison with preoperative, *P* < 0.05; ^#^Comparison with immediately after surgery, *P* < 0.05; ^&^Comparison with 6 h after surgery, *P* < 0.05; ^△^Comparison with 12 h after surgery, *P* < 0.05.

**Table 5:** Comparison of adverse reactions (*n*, %).

Group	Restlessness	Low blood pressure	Tachycardia	Bradycardia	Nausea and vomiting	Incidence of adverse reactions
Combined anesthesia group (*n* = 142)	7(4.93)	2(1.41)	4(2.82)	5(3.52)	2(1.41)	21 (14.79)
The control group (*n* = 143)	17(11.89)	11(7.69)	10(6.99)	9(6.29)	8(5.59)	55 (38.46)
*x* ^2^	—	—	—	—	—	20.418
*P*	—	—	—	—	—	＜0.001

**Table 6:** Differences in the PSQI scores at different time points (score, $\bar{x}$ ± *s*).

Group	24 h after surgery	48 h after surgery	7 d after surgery
Combined anesthesia group (*n* = 142)	12.35 ± 2.72	8.64 ± 1.95^∗#^	4.74 ± 1.32^∗#^
The control group (*n* = 143)	13.04 ± 2.86	9.73 ± 2.11^∗#^	6.38 ± 1.59^∗#^
*T*	−2.087	−4.528	−9.470
*P*	0.038	<0.001	<0.001
Between groups	*F* = 5.551, *P*=0.000		
Different points in time	*F* = 5.288, *P*=0.000		
Between groups *·* different time points	*F* = 4.837, *P*=0.000		

*Note.* ^*∗*^ *P* < 0.05 compared with 24 h after surgery, *P* < 0.05; ^#^*P* < 0.05 compared with 48 h after surgery.

## Data Availability

The simulation experiment data used to support the findings of this study are available from the corresponding author upon request.
